# Study on the Interactive Factors between Physical Exercise and Mental Health Promotion of Teenagers

**DOI:** 10.1155/2022/4750133

**Published:** 2022-01-25

**Authors:** Zhifeng Guo, Yiying Zhang

**Affiliations:** ^1^Department of Sports, Kunming University of Science and Technology, Kunming, Yunnan 650500, China; ^2^Youth League Committee, Kunming University of Science and Technology, Kunming, Yunnan 650500, China

## Abstract

Adolescence is a key period of growth in life, and the psychological development of teenagers in this period is in a stage of rapid maturity without maturity, with distinct characteristics of self-contradiction. People's in-depth understanding of the concept of mental health has prompted people to have a new understanding of the function of physical exercise, trying to make an in-depth study of the function of physical exercise. Teenagers are considered to be the main force for the future development of our society, so in the process of educating teenagers, we should not only pay attention to the exercise of physical quality but also pay attention to the education of psychological quality. With the rapid development of modern society and science and technology, human life is becoming more and more prosperous, and people have to face various conflicts and troubles. The faster pace of life makes people face more pressure. In this paper, the interaction between adolescent physical exercise and mental health factors is discussed, and the promotion effect of physical exercise on college students' mental health is analyzed, so as to provide theoretical basis for further improving adolescent mental health.

## 1. Introduction

As an important concept of health, mental health is closely related to our life, social economy, and culture. People's in-depth understanding of the concept of mental health prompted people to have a new understanding of the function of physical exercise, trying to conduct in-depth research on the function of physical exercise [1]. Mental health means that individuals can adapt to the development of the environment and respond to cognitive emotions. The behavior is put in a positive state, and normal adjustment ability is maintained [2]. The basic characteristics of mental health are to be able to control oneself with self-control, to view the influence of the external environment with a correct attitude, and to keep psychological balance and coordination [3]. For young college students, physical health education and mental health education are equally important, so in physical education, we should not only focus on physical fitness exercise but also, through physical exercise, take appropriate ways to strengthen the mental health education of young college students, so as to deeply tap the intrinsic value of physical education [4]. Because teenagers are in the growth period and have limited ability to bear psychological problems, they become the important victims of various psychological diseases, which is the most volatile stage in the growth process. The unstable factors in the growth process of adolescents include genetic factors, malnutrition, and acute infection, which often prevent weight gain or loss. Chronic infection affects the growth of weight and height at the same time. Endocrine diseases (such as hypothyroidism) have a more prominent impact on growth and development. In the context of traditional exam-oriented education, students' growth is often accompanied by great learning pressure, especially adolescent students. Many of them have entered the middle school stage. Compared with the learning content of primary school, the subjects of junior and senior high school are more and more difficult [5]. During this period, thinking, emotion and will gradually form and develop, and become mature. Various psychological contradictions and conflicts, such as emotion and reason, ideal and reality, independence and dependence, desire for communication and psychological closure, crisscross and even constitute psychological obstacles [6].

As a group with higher education level, the development of college students affects the direction of China's economic and cultural development to a certain extent. They can provide a solid talent foundation for the rapid development of the country and are also the key groups trained by the National Education Department [7]. With the rapid development of modern society and science and technology, human life is increasingly prosperous, people have to face all kinds of conflicts and troubles, and faster pace of life makes people face more pressure. With fierce social competition and complex social relations, people often feel anxious, tired and uneasy. More and more people realize that fear, anxiety, anger, and depression will affect personal health [8]. Good sports lifestyle can improve the ability of teenagers from different aspects. At present, it is particularly important to guide teenagers to establish and develop a good sports lifestyle [9]. There is no unified view on the possible mechanism of psychological benefits produced by physical exercise. Whether different psychological benefits have different physiological mechanisms remains to be explored [10]. This paper discusses the interaction between physical exercise and mental health factors of teenagers and analyzes the promoting effect of physical exercise on mental health of college students, so as to provide theoretical basis for further improving mental health of teenagers.

## 2. Interaction between Sports Lifestyle and Mental Health Benefits of Teenagers

Through the investigation and analysis of the promoting factors of teenagers' mental health, the four dimensions of promoting their mental health in physical exercise are sense of behavior control, behavior intention, behavior habit, and emotional experience. Regular physical exercise can release the excess energy of the human body, reduce the degree of anxiety and depression of teenagers, relieve tension, promote interpersonal relations, improve self-esteem and self-confidence, and promote the level of mental health. Sports lifestyle refers to the stable form and behavior characteristics of all sports activities that meet the multi-level needs guided by certain values of individuals, groups, or all members of the society under the constraints of certain social objective conditions. Interpersonal relationship is an important part of mental health education. Modern young college students are basically only children. In the process of growing up, they get comprehensive care from their families. Therefore, it is easy to lead them to lack of team consciousness and unwilling to communicate with others. Through physical exercise, we can cultivate the interpersonal skills of young college students. Physical exercise refers to the physical activities to improve physical fitness and shape a good body. Activities are more diversified, such as ball games, water sports, track, and field events, mainly individual or collective activities. Physical exercise is beneficial to physical and mental health. Physical health and mental health depend on each other. Physical and mental health is a unity. Contemporary teenagers have too much learning pressure and less spare time. On weekends, teenagers are occupied with a lot of time by various classes and have no time to participate in sports activities [11]. Teenagers lack interest in participating in sports activities, are occupied by games and electronic products in their spare time, and lack a correct understanding of their own physique. Physical exercise can not only improve the physical quality of individuals but also improve the communication ability between individuals and others and bring diversified fun to life and promote individuals to have better psychological quality.  Table 1 shows the survey of psychological training program.

Physical exercise can not only help students know more about their special skills, make proper and objective evaluations of their abilities, personalities, and advantages, and not put forward harsh and presumptuous delusions but also develop their potential, experience the value of their existence, and correct their self-awareness. Some students may always be in an advantageous position in academic achievement, so they will have a sense of superiority and pride in psychology. However, if they encounter setbacks, they will experience a great psychological blow and cannot accept the reality. Therefore, it is necessary to guide young students psychologically and realize that success and failure are things that must be experienced in life, and there is no smooth road. With the improvement of people's cognitive level, mental health is also an important criterion for judging health. Therefore, in modern times, people's cognition of health should include both physical health and mental health. Physical health lays the foundation for the development of life, and mental health better guides the development towards positive health [12]. At the same time, family education is particularly important. Family education with different backgrounds has different influences on teenagers' character and mood and also affects the formation of their sports lifestyle. Good family education will help teenagers form better habits of participating in sports activities, while poor family education will hinder the formation of teenagers' sports lifestyle. Mental health means that an individual can live in harmony with the society, can be in good self-condition, have the ability to reduce problem behaviors and resist mental illness, and can be in the best state of mind.

In the process of physical exercise, you will experience all kinds of successes and failures, and you will appreciate joy and pain in the process of exercise. Rich emotional experience is conducive to cultivating students' healthy emotions, so that they can adjust their emotions and face failure calmly. When students contact and communicate with other students directly or indirectly in sports activities, they will have a sense of closeness and gain the ability to communicate correctly with other students. Therefore, physical exercise is conducive to coordinating interpersonal relationships and enables people in the same collective to learn to care for each other and understand and help others, thus forming the habit of communicating and cooperating with others. Physical exercise can prevent the occurrence of mental diseases of young students and make them mentally healthy. When students have psychological problems, if they can get timely guidance and solution, they can resolve the psychological problems in the bud. Teenagers can exercise, shape, and enhance their self-confidence when participating in sports such as sports dance, aerobics, and yoga, especially in enhancing the self-confidence of girls. First of all, athletes should understand the goals and tasks of sports training from an early age, so that the team members can consciously mobilize their enthusiasm, persistence, and tenacity in training. Secondly, the objectives and requirements of coaches should be trained according to the sports ability of each team member.

## 3. Measures of Physical Exercise to Promote the Mental Health Development of Young Students

### 3.1. Guiding Students to Actively Participate in Physical Exercise

Proper physical exercise for college students can not only strengthen their physical fitness but also effectively ensure their better mental health, which is of great significance to the cultivation of talents in China. In the teaching of physical education theory, students are taught the knowledge of mental health education in various ways, so that students can understand that true health includes physical health, mental health, and certain social adaptability, all of which are indispensable. At present, with the deepening of education reform, college students' physical exercise has become an important task of education reform. Therefore, strengthening physical exercise and improving college students' mental health quality are not only the task entrusted by the times but also the fundamental requirement of College Students' self-development. Teachers should publicize and guide students to take an active part in physical exercise, cultivate their awareness of physical exercise, and achieve the purpose of strengthening their physique and enjoying their body and mind in sports.

Physical exercise can constantly cultivate their good self-discipline ability and improve students' temperament, which plays a positive role in enhancing their personal charm. Therefore, in view of the sports facilities of the school, the relevant departments of the school should actively improve and optimize, give students more choices of physical exercise, and let them keep moving forward on the road of enhancing their personal charm. The interactive relationship of students' social development is shown in Figure 1.

Teachers should make full use of the advantages of sports activities in physical education class and ask students to take part in various physical exercises according to their various unhealthy psychological states, so as to strengthen the willpower training of young students and enhance their self-confidence. By organizing many physical exercises with different contents and forms, teachers can enrich students' spare time, cultivate students' sentiment, establish good interpersonal relationships, and make students develop well physically and mentally. Colleges and universities should actively carry out competitions in various sports activities, combine with social organizations, carry out sports competitions and bodybuilding competitions, and give spiritual and material rewards to those who perform best [13]. Activities in this situation can not only make students connect with the society but also make them better aware of the importance of building a strong body to enhance their personal charm and mental health. In the teaching of physical education theory, students are taught the knowledge of mental health education in various ways, so that students can understand that true health includes physical health, mental health, and certain social adaptability, all of which are indispensable.

### 3.2. Making a Feasible Physical Education Plan

Teenagers' original psychological level is gradually improved when they improve their sports level or beat their opponents. That is to say, the contradiction between the new needs of sports and the original psychological level promotes the development of psychology. School physical education teachers should make full use of physical education classroom time to cultivate their good interest in physical exercise and give them guidance on physical exercise to deepen their correct understanding of physical exercise. They can also use rich teaching contents and diversified teaching methods to stimulate their interest in learning. Sports also contribute to self-education. On the basis of a correct understanding of self, one will consciously or unconsciously correct one's own understanding and behavior, cultivate and improve the psychological quality and various abilities needed by society, and make himself a person who can better meet the needs and adapt to society. To make students psychologically healthy, teachers should be psychologically healthy first. Therefore, schools should educate physical education teachers on mental health knowledge, so that they can master the related knowledge of adolescent students' mental health, psychological consultation, and mental health care and master specific operating principles.  Figure 2 shows the system structure of special sports psychological prevention method.

Physical exercise is generally characterized by fierce confrontation and strong competitiveness. When teenagers take part in physical exercise, they are always accompanied by strong emotional experience and obvious will. Therefore, physical exercise helps to cultivate young people's courage, tenacity, perseverance, and ideological style of overcoming difficulties, as well as collectivism and patriotism. Teachers should pay attention to students' physical exercise in physical education, not only the education of physical theory but also pay due attention to physical exercise in classroom teaching, such as organizing group games or sports games, so as to strengthen students' physical exercise. In addition, teachers need to guide students' physical exercise, so that students' physical exercise can produce better results and improve students' physical fitness.

## 4. Conclusions

For modern college students, they lack exercise in self-reliance, willpower, emotional processing, interpersonal relationship, and so on. In the face of setbacks, because they cannot face up to themselves, they will have serious mental illness, which is not conducive to the healthy growth of students. Physical exercise is an important way to train young students to develop in an all-round way. Physical exercise has a positive impact on strengthening college students' psychological quality, improving their ability to resist pressure and solving social problems. Physical exercise can improve young students' intelligence and promote their health, and it is also an important factor affecting their mental health. Regular physical exercise can make them feel comfortable physically and mentally. Schools should educate physical education teachers on mental health knowledge, so that they can master the related knowledge of adolescent students' mental health, psychological counseling, and mental health care and master specific operating principles. Teenagers, as the future of society, should not only cultivate their good habits in study but also develop their abilities in many ways. Teenagers' physique is declining, so we should pay attention to teenagers' physique problems, train them to develop a good sports lifestyle, explore suitable sports, carry out reform and innovation constantly, attract teenagers' participation, and cultivate their interest in sports.

## Figures and Tables

**Figure 1:** Interactive relationship of students' social development.

**Figure 2:** System structure of psychological prevention methods for special sports.

**Table 1:** Survey of psychological training plans.

	Number of people	Proportion (%)
Make a systematic psychological training plan	28	7
Arrange according to experience	372	93

## Data Availability

The data used to support the findings of this study are included within the article.
